# Both Food Restriction and High-Fat Diet during Gestation Induce Low Birth Weight and Altered Physical Activity in Adult Rat Offspring: The “Similarities in the Inequalities” Model

**DOI:** 10.1371/journal.pone.0118586

**Published:** 2015-03-04

**Authors:** Fábio da Silva Cunha, Roberta Dalle Molle, André Krumel Portella, Carla da Silva Benetti, Cristie Noschang, Marcelo Zubaran Goldani, Patrícia Pelufo Silveira

**Affiliations:** 1 Programa de Pós-Graduação da Saúde da Criança e do Adolescente, Departamento de Pediatria, Faculdade de Medicina, Hospital de Clínicas de Porto Alegre, Universidade Federal do Rio Grande do Sul, Porto Alegre, Rio Grande do Sul, Brazil; 2 Departamento de Pediatria, Universidade Federal de Ciências da Saúde de Porto Alegre, Porto Alegre, Rio Grande do Sul, Brazil; Monash University, AUSTRALIA

## Abstract

We have previously described a theoretical model in humans, called “Similarities in the Inequalities”, in which extremely unequal social backgrounds coexist in a complex scenario promoting similar health outcomes in adulthood. Based on the potential applicability of and to further explore the “similarities in the inequalities” phenomenon, this study used a rat model to investigate the effect of different nutritional backgrounds during gestation on the willingness of offspring to engage in physical activity in adulthood. Sprague-Dawley rats were time mated and randomly allocated to one of three dietary groups: Control (Adlib), receiving standard laboratory chow ad libitum; 50% food restricted (FR), receiving 50% of the ad libitum-fed dam’s habitual intake; or high-fat diet (HF), receiving a diet containing 23% fat. The diets were provided from day 10 of pregnancy until weaning. Within 24 hours of birth, pups were cross-fostered to other dams, forming the following groups: Adlib_Adlib, FR_Adlib, and HF_Adlib. Maternal chow consumption and weight gain, and offspring birth weight, growth, physical activity (one week of free exercise in running wheels), abdominal adiposity and biochemical data were evaluated. Western blot was performed to assess D2 receptors in the dorsal striatum. The “similarities in the inequalities” effect was observed on birth weight (both FR and HF groups were smaller than the Adlib group at birth) and physical activity (both FR_Adlib and HF_Adlib groups were different from the Adlib_Adlib group, with less active males and more active females). Our findings contribute to the view that health inequalities in fetal life may program the health outcomes manifested in offspring adult life (such as altered physical activity and metabolic parameters), probably through different biological mechanisms.

## Introduction

There is considerable evidence to support the view that physical activity is a modifiable behavior, which can benefit overall health by reducing mortality [1–3], preventing cardiovascular diseases [4,5], and improving psychological well-being and quality of life [6–8]. Nevertheless, the World Health Organization estimates that 60% to 85% of the population in developed and transitional countries is physically inactive [9]. Ethnicity [10,11], sex and age [11–13], birth weight [14] and birth order [15] are some of the biological determinants of physical activity. Social determinants of physical activity include parental education, socioeconomic status [10,11,16], and neighborhood safety [17,18], among others.

We have previously shown in humans that individuals with normal birth weight and higher levels of education are as likely as low-birth-weight individuals with lower levels of education to be physically inactive [19]. This particular scenario, in which extremely unequal backgrounds coexist in a complex manner promoting similar health outcomes in adulthood, was called the “Similarities in the Inequalities” model [20]. In our previous study [19], both biological characteristics and social factors were correlated with physical activity in adulthood, indicating that individuals of opposed backgrounds may converge to similar health outcomes even when they face unequal conditions during their life course. Such a scenario is believed to occur mainly in countries with high levels of social inequality.

In Latin America and the Caribbean, while large segments of the population are affected by hunger and undernutrition, malnutrition, in the form of overeating, is increasing daily. This profile reflects the large inequality of income distribution and social protection in these countries, where extremely poor populations live side by side with groups enjoying the benefits of wealth and economic development [21].

Although socioeconomic status cannot be measured for animals, animal models are able to capture many components and correlates of socioeconomic status, including prenatal factors, such as maternal nutrition, stress, and disease exposure during pregnancy, as well as postnatal variations, such as maternal behavior and environmental stimulation [22,23]. Recent studies have proposed that different methods of inducing maternal malnutrition during pregnancy (including both maternal undernutrition and overnutrition) are able to alter postnatal phenotype and the development of metabolic disease in the adult offspring [24]. This suggests that different nutritional insults act on a limited set of common genes or gene pathways, leading to the same adult phenotype, what some authors have termed the ‘‘gatekeeper hypothesis” [25].

In view of the above considerations, our objective was to investigate the effect of different nutritional backgrounds affecting fetal growth during gestation on the willingness of offspring to engage in physical activity in adulthood. Based on the “Similarities in the Inequalities” model, in which privileged and underprivileged individuals (with opposed perinatal backgrounds) had similar health behaviors in adulthood, we hypothesized that an animal model, considering food abundance and scarcity as extremes of inequality during gestation, could potentially mimic the “similarities in the inequalities” phenomenon previously described in humans [19].

## Materials and Methods

### Ethical approval

All animal procedures were approved by the Institutional Ethics Committee of Hospital de Clínicas de Porto Alegre (GPPG/HCPA, project number 11–0053) and followed national and international guiding principles for research involving animals, including the Brazilian Law No. 11,794 (2008).

### Rats mating and maternal diet

Virgin Sprague-Dawley rats, approximately 80 days old, were time mated at our animal facility after daily vaginal smearing. Pregnancy was confirmed on day 1 by the presence of sperm in the vaginal smear. During pregnancy, the rats were housed individually in Plexiglas cages (49×34×16 cm) and maintained under a standard light-dark cycle (lights on 0900–1900 h) in a temperature-controlled room (22 ± 2°C). The cages were cleaned once a week, and food and water were provided ad libitum. At 10 days of gestation, dams were randomly allocated to one of three dietary groups: (i) control (Adlib) (n = 21), receiving standard laboratory chow ad libitum (2.95 kcal/g, 15% protein, 12% fat, 73% carbohydrate); (ii) 50% food restricted (FR) (n = 14) (based on the intrauterine growth restriction model described by Desai et al. [26]), receiving 50% of the ad libitum-fed dam’s intake (determined after quantification of the mean daily intake of the control group); or (iii) high-fat diet (HF) (n = 12), receiving a diet containing 4.59 kcal/g, 47% carbohydrate, 25% protein, 23% fat, and 5% fiber. The diets were provided from day 10 of pregnancy until weaning.

### Offspring

Within 24 hours of birth, all pups were weighed and the litters were culled to eight pups (four males and four females). The pups from each litter were cross-fostered to other dams, forming the following groups considering the biological/adoptive dam (gestation/lactation maternal) diet: Adlib_Adlib, FR_Adlib, FR_FR, Adlib_FR, HF_Adlib, HF_HF, and Adlib_HF. In order to examine the “similarities in the inequalities” phenomenon in this animal model, the analyses described in this study focus on only three groups: Adlib_Adlib, as the reference group, and FR_Adlib and HF_Adlib, representing the extremes of nutritional inequality during fetal life (i.e., maternal undernutrition and overnutrition, respectively). Data from the other groups were redirected to a different research project.

To avoid biases regarding running abilities and metabolism due to handling [27,28], pups were left undisturbed with their adoptive dams until weaning. On postnatal day 21, pups were weaned and housed with pups of the same sex from the same litter (3–4 rats/cage). All animals were fed standard laboratory chow and water ad libitum and maintained in the same controlled conditions as described above, except for the light-dark cycle (lights on 0700–1900 h). From day 21 onwards, body weight was measured once a week at the time of cage cleaning using a digital scale to the nearest 0.01 g. No more than two pups of the same sex per litter were used for the same experiment.

### Physical activity

After completing 60 days of life (which corresponds to a young adult in humans), the rats were isolated for one week and then housed individually in cages with running wheels (20 cm diameter) where they could exercise freely for seven days. All wheels had sensors connected to digital counters, which continuously recorded the rats’ total and partial activity every minute. The female estrous cycle was not evaluated because the period of exercise monitoring (seven consecutive days) included all phases of the estrous cycle.

### Tissue collection and biochemical analysis

Twenty-four hours after the end of exercise monitoring, the animals were decapitated after 4 hours of fasting. The two major portions of abdominal fat (gonadal and retroperitoneal adipose tissue depots) were dissected and weighed. Data on abdominal fat was expressed as percentage of body weight. Glucose, total cholesterol, high density lipoprotein (HDL) and triglyceride (TG) plasma levels were determined by the biochemists of the clinical laboratory at our hospital using a standard enzymatic colorimetric method, which determines with the aid of a color reagent the concentration of a chemical compound in a solution undergoing an enzymatic reaction. Plasma insulin levels were quantified at our laboratory by ELISA, using commercial reagents (Rat/Mouse Insulin ELISA Kits). The Homeostasis Assessment Model- insulin resistance (HOMA-IR) was calculated using the following formula: insulin (μU/mL) × glucose (mmol/L)/22.5.

The brains were also dissected, flash frozen in isopentane, and stored at -80°C. For dissection of the dorsal striatum, frozen brains were warmed to -20°C and coronal sections of 0.25 cm were cut. The dorsal striatum was identified with the aid of an atlas [29] and punches of 1 mm diameter were made to isolate this brain region. The extracts obtained were processed for Western blot analysis as described below.

### Western Blot

Dorsal striatum samples were homogenized in cytosolic extraction buffer with protease (Protease Inhibitor Cocktail) and phosphatase inhibitors (PhosSTOP Phosphatase Inhibitor Cocktail Tablets). The samples were centrifuged at 3000 rpm for 10 minutes at 4°C for extraction of the cytosolic fraction. After that, an additional centrifugation at 13000 rpm for 30 minutes at 4°C was performed to obtain a more purified cytosolic fraction. Part of the supernatant (2 μL) was used to quantify total protein, which was determined with a bicinchoninic acid (BCA) kit using bovine serum albumin as a standard. Supernatant containing 40 μg of protein was incubated with lithium dodecyl sulfate (LDS) and dithiothreitol (DTT) at 99°C for 3 minutes. These samples and a molecular weight standard (MagicMark) were loaded on 4–12% polyacrylamide gradient gels, subjected to electrophoresis, and then transferred to a nitrocellulose membrane. The blots were blocked in Tris-buffered saline containing 10% nonfat milk and 1% Tween-20. The membranes were incubated overnight with the primary antibody (anti-dopamine D2 receptor antibody, 1:1,000). The next day, the membranes were incubated for 1 hour with the secondary antibody (anti-rabbit IgG antibody, 1:2,000), then developed (Amersham Hyperfilm ECL) and visualized using the enhanced chemiluminescence (ECL) Western blotting analysis system. Western blot band intensity was quantified by densitometric analysis using a free software developed by the National Institutes of Health. Results were expressed as the ratio between the protein of interest and β-actin (1:1,000).

### Statistical analysis

Data were tested for normality using the Shapiro-Wilk test. Gestational data were analyzed using generalized estimating equations (GEE) with group and time as independent variables (or factors) and litter size as a covariate. Litter size was analyzed by one-way ANOVA followed by Tukey’s post hoc test, and neonatal mortality by the chi-square test. Birth weight data were analyzed using GEE with group and sex as factors, adjusted for litter size. The analyses were followed by Bonferroni multiple comparison test when appropriate. A GEE analysis was used to evaluate the rats from the same litter as a block so that variations within each rat could be considered in the model.

Weight gain during development was analyzed separately by sex using GEE with group and time as independent variables. Physical activity was also analyzed using GEE with group and time as factors. For the purpose of analysis, data were grouped into intervals of 4 hours over the day [30], as follows: interval 1 (07:00–10:59 AM); interval 2 (11:00 AM-02:59 PM); interval 3 (3:00–6:59 PM); interval 4 (7:00–10:59 PM); interval 5 (11:00 PM-02:59 AM); and interval 6 (3:00–6:59 AM). Because sex differences in wheel-running activity were extremely high (over a 100-times difference) and the comparison between males and females in this outcome was not a primary objective of the study, these data were then analyzed separately by sex. The analyses were followed by Bonferroni multiple comparison test when appropriate.

Longitudinal data were analyzed using GEE because this method allows the evaluation of continuous data even when the assumptions of normality and sphericity are violated [31]. In addition, even when data are missing for a specific item in an individual, it is possible to include all individuals, thus avoiding selection bias [32]. Also, GEE was used instead of repeated-measures ANOVA because it requires a smaller sample size to show the same effect size with 80% power [33].

Two-way ANOVA was used to analyze abdominal fat deposition and biochemical measurements, with group and sex as factors, followed by Tukey’s post hoc test when appropriate and also using the three models described above. Because TG levels were asymmetric, the data were log transformed (and expressed as median and interquartile range) and then analyzed by two-way ANOVA.

The Student t test was used to analyze Western blot data. The analyses were performed separately by sex and only samples from the same nitrocellulose membrane were compared (Adlib_Adlib males vs. FR_Adlib males / Adlib_Adlib males vs. HF_Adlib males / Adlib_Adlib females vs. FR_Adlib females / Adlib_Adlib females vs. HF_Adlib females).

All statistical analyses were performed using the Statistical Package for the Social Sciences (SPSS), version 18.0. The level of significance was set at p < 0.05 for all statistical tests.

## Results

### Gestational data

The GEE analysis of dam body weight during gestation revealed a group vs. time interaction (Wald = 402.05; gl = 8; p<0.001; n = 9–17/group). At 13 days of gestation, HF dams were heavier than FR dams (Bonferroni post hoc test, p<0.001). On gestation days 16, 18 and 21, HF and Adlib dams were heavier than FR dams (Bonferroni post hoc test, p<0.001). Food intake during gestation was also analyzed by GEE and a group vs. time interaction was found (Wald = 23.07; gl = 8; p = 0.003; n = 8–17/group). As expected, because of the protocol design, FR dams consumed fewer calories than HF and Adlib dams throughout pregnancy (Bonferroni post hoc test, p<0.05). No differences were found between HF and Adlib dams (Bonferroni post hoc test, p>0.05) (Fig. 1A and B).

**Fig 1:** Body weight gain (A) and food intake in calories (B) throughout gestation. Data are expressed as mean ± SEM. Analyses adjusted for litter size. (A) GEE showed a group vs. time interaction (p<0.001). *Bonferroni post hoc test (p<0.001), HF > FR. **Bonferroni post hoc test (p<0.001), HF and Adlib > FR. (B) GEE showed a group vs. time interaction (p = 0.003). *Bonferroni post hoc test (p<0.05), HF and Adlib > FR.

Using GEE to compare the relationship between weight gain and caloric intake during gestation [(final weight − baseline weight)/total caloric intake in the period] during three gestational periods after the beginning of the dietary interventions (period 1: day 10 to 13; period 2: day 14 to 18; period 3: day 19 to 21), we found an interaction between group and time (Wald = 20.404; gl = 4; p<0.0001; n = 12/group). The Bonferroni post hoc test showed that FR dams gained less weight per calorie than HF and Adlib dams during period 1 (FR: 0.06±0.02; HF: 0.06±0.009; Adlib: 0.05±0.007) and 2 (FR: 0.005±0.013; HF: 0.11±0.008; Adlib: 0.12±0.006) (p<0.0001 for all comparisons). There were no differences between HF and control dams. These analyses were adjusted for the number of pups per dam.

The dietary intervention during gestation did not affect litter size (Adlib: 11.89±2.00; FR: 9.64±3.9; HF: 10.78±2.49; one-way ANOVA, p = 0.118; Tukey’s HSD test, p>0.05). There was no difference in the percentage of males (Adlib: 52.2%; FR: 43.0%; HF: 52.1%; chi-square test, p = 0.296) and females (Adlib: 47.8%; FR: 57.0%; HF: 47.9%; chi-square test, p = 0.296) between groups. However, neonatal mortality was higher in the HF group (Adlib: 6.3%; FR: 3.1%; HF: 14.6%; chi-square test, p = 0.010).

### Birth weight

The GEE analysis of birth weight revealed a group vs. sex interaction (Wald = 6.681; gl = 2; p = 0.035; n = 62–126/group), adjusted for litter size. In both sexes, pups born to dams exposed to FR (Bonferroni post hoc test, p<0.0001) and to HF (Bonferroni post hoc test, p<0.018) had a lower birth weight than the offspring of controls (Fig. 2), an example of the “similarities in the inequalities” effect. FR and HF did not differ from each other (Bonferroni post hoc test, p = 0.722). As expected, males weighed more than females in the Adlib group (Bonferroni post hoc test, p<0.006), but this sex difference was not observed in the other two groups (Bonferroni post hoc test, p = 0.550 for FR and p = 0.090 for HF).

**Fig 2:** Birth weight (g) in Adlib, FR, and HF groups. Data are expressed as mean ± SEM. Analysis adjusted for litter size. Males: n = 37–128/group, females: n = 34–117/group. GEE showed a sex vs. group interaction (p = 0.035). * FR and HF males and females weigh less than Adlib males and females. Bonferroni post hoc test: FR vs. Adlib (p<0.0001), HF vs. Adlib (p = 0.018).

### Weight gain during development

Fig. 3 shows body weight throughout life separately by sex. In males, GEE showed a group vs. time interaction (Wald = 100.019; gl = 12; p<0.0001), because of a subtle difference between groups at weeks 6 and 7 (FR_Adlib at week 7 had the same body weight as Adlib_Adlib and HF_Adlib at week 6). Nevertheless, there was no difference between groups within each week (Bonferroni post hoc test, p>0.05). A time effect alone was also observed (Wald = 10515.121; gl = 6; p<0.0001). In females, only a time effect was observed (Wald = 17546.22; gl = 6; p<0.0001), reflecting the body weight gain throughout life in all groups. There was no group effect (Wald = 0.630; gl = 2; p = 0.730) or group vs. time interaction (Wald = 19.224; gl = 12; p = 0.083).

**Fig 3:** Body weight during development (g) in males (A) and females (B). Data are expressed as mean ± SEM. Males: n = 13–39/group, females: n = 13–42/group. (A) GEE showed a group vs. time interaction (p<0.001). (B) GEE showed a time effect (p<0.001).

### Physical activity

Figs. 4 and 5 illustrate the results of physical activity separately for males and females, respectively. Figs. 4A and 5A show the mean number of wheel turns made by the rats, considering the seven days of physical activity. Figs. 4B, 4C, 4D, 5B, 5C and 5D show the actograms that demonstrate the wheel-running activity rhythms per day.

**Fig 4:** Number of wheel turns (physical activity) by males. Data are expressed as mean ± SEM (A) and plotted as actograms: (B) Adlib_Adlib, (C) FR_Adlib, (D) HF_Adlib. (A) * Extreme groups (FR_Adlib and HF_Adlib) were less active than the reference group (Adlib_Adlib) (GEE, p<0.001; Bonferroni post hoc test, p<0.05; n = 7–9/group). (B) (C) (D) Actograms: wheel-running activity rhythms are shown as bars representing 15 minutes. Time of the day is indicated on the X axis and number of days on the Y axis. Horizontal white and black bars above the actograms indicate the duration of the light and dark phases, respectively, of the light-dark cycle.

**Fig 5:** Number of wheel turns (physical activity) by females. Data are expressed as mean ± SEM (A) and plotted as actograms: (B) Adlib_Adlib, (C) FR_Adlib, (D) HF_Adlib. (A) * Extreme groups (FR_Adlib and HF_Adlib) were more active than the reference group (Adlib_Adlib) (GEE, p<0.001; Bonferroni post hoc test, p<0.05; n = 7–9/group). (B) (C) (D) Actograms: wheel-running activity rhythms are shown as bars representing 15 minutes. Time of the day is indicated on the X axis and number of days on the Y axis. Horizontal white and black bars above the actograms indicate the duration of the light and dark phases, respectively, of the light-dark cycle.

When examining the “similarities in the inequalities” effect on physical activity, the GEE analysis showed an interaction between group and time intervals (Wald = 48.745; gl = 10; p<0.0001, n = 7–9/group), as well as a group effect alone (Wald = 12.208; gl = 2; p = 0.002) and a time effect alone (Wald = 71.504; gl = 5; p<0.0001) in males. The results of the Bonferroni post hoc test for this interaction also indicated a “similarities in the inequalities” effect on the willingness to engage in exercise, in which the extreme groups (FR_Adlib and HF_Adlib) showed a significantly lower wheel-running activity level than the Adlib_Adlib (reference) group in interval 3 (15:00–18:59 h) (Adlib_Adlib vs. FR_Adlib, p = 0.004; Adlib_Adlib vs. HF_Adlib, p = 0.020), almost reaching statistical significance in interval 6 (03:00–06–59 h) (Adlib_Adlib vs. FR_Adlib, p = 0.055; Adlib_Adlib vs. HF_Adlib, p = 0.014) (Fig. 4A-D). Extreme groups differed from each other only in interval 5 (23:00–02:59 h), in which the FR_Adlib group was more active than the HF_Adlib group (p<0.0001). There were no differences between groups in other time intervals.

In females, there was also an interaction between group and time (Wald = 45.830; gl = 10; p<0.001, n = 7–9/group), as well as a group effect alone (Wald = 6.196; gl = 2; p = 0.045) and a time effect alone (Wald = 101.618; gl = 5; p<0.001). The analysis using the Bonferroni post hoc test also showed the “similarities in the inequalities” effect, in which the extreme groups (FR_Adlib and HF_Adlib) were significantly more active than the reference group (Adlib_Adlib) in interval 4 (19:00–22:59 h) (Adlib_Adlib vs. FR_Adlib, p = 0.005; Adlib_Adlib vs. HF_Adlib, p<0.0001) (Fig. 5A-D). There were no differences between groups in other time intervals.

### Abdominal fat deposition

Table 1 describes the results for abdominal fat. There was no difference between groups [two-way ANOVA, F (2, 82) = 0.915, p = 0.405] or sexes [two-way ANOVA, F (1, 82) = 1.191, p = 0.278], as well as no group vs. sex interaction [two-way ANOVA, F (2, 82) = 0.914, p = 0.405].

**Table 1:** Abdominal fat deposition expressed as a percentage of total body weight.

**Group/sex**	**Adlib_Adlib (n = 18–21)**	**FR_Adlib (n = 13–15)**	**HF_Adlib (n = 10–11)**
Males	1.77±0.53	2.07±0.62	1.68±0.68
Females	3.18±0.49	2.33±0.58	1.62±0.71

Data are expressed as mean ± SEM. No effects of group, sex or interactions were observed. See text for details.

### Biochemical measurements

Tables 2 and 3 show the results of biochemical measurements in males and females respectively. Regarding glucose levels, a group effect was observed [two-way ANOVA, F (2, 44) = 8.061, p = 0.001], in which the FR_Adlib group had increased glucose levels in relation to the HF_Adlib (Tukey’s test, p = 0.001) and Adlib_Adlib (Tukey’s test, p = 0.008) groups. There was no sex effect [F (1, 44) = 2.058, p = 0.158] or group vs. sex interaction [F (2, 44) = 1.569, p = 0.220]. Similar results were observed for insulin levels with a group effect [two-way ANOVA, F (2, 32) = 5.55, p = 0.009], in which FR_Adlib had increased insulin levels in relation to Adlib_Adlib (Tukey’s test, p = 0.010), but with no difference in relation to HF_Adlib (Tukey’s test, p = 0.166). No sex effect [F (1, 32) = 2.068, p = 0.160] or group vs. sex interaction were observed [F (2, 32) = 2.592, p = 0.091]. The analysis of HOMA-IR revealed only a group effect [two-way ANOVA, F (2, 32) = 7.98, p = 0.002], in which FR_Adlib had increased HOMA-IR in relation to Adlib_Adlib (Tukey’s test, p = 0.002) and HF_Adlib (Tukey’s test, p = 0.032). There was no sex effect [F (1, 32) = 1.329, p = 0.257] or group vs. sex interaction [F (2, 32) = 2.128, p = 0.136].

**Table 2:** Biochemical measurements in males.

**Measurement**	**Males (n = 6–9/group)**		
	***Adlib_Adlib***	**FR_*Adlib***	**HF_*Adlib***
Glucose (mg/dL)	135.8±3.6 ^x^	142.1±3.8 ^y^	126.5±3.8 ^x^
Insulin (ng/mL)	0.90±0.15 ^x^	2.03±0.32 ^y^	1.34±0.22 ^x^, ^y^
HOMA-IR	0.31±0.05 ^x^	0.72±0.11 ^y^	0.41±0.07 ^x^
Total cholesterol (mg/dL)	81.3±4.6 ^x^	94.8±4.9 ^y^	91.6±4.9 ^x^, ^a^
HDL cholesterol (mg/dL)	25.0±1.5 ^x^	30.5±1.6 ^y^	27.5±1.6 ^x^
Triglycerides (mg/dL)	153.0±80.5 ^a^	114.5±28.5 ^a^	140.0±85.8 ^a^

Data are expressed as mean ± SEM except for triglycerides (levels were asymmetric and therefore data was log transformed and expressed as median and interquartile range). ^x,y, a,b^ Values labeled with the same letter are statistically similar and different letters refer to statistical difference by Tukey *post hoc*.

^x,y^ groups comparison

^a,b^ sex comparison (compare tables 2 and 3).

**Table 3:** Biochemical measurements in females.

**Measurement**	**Females (n = 6–10/group)**		
	***Adlib_Adlib***	**FR_*Adlib***	**HF_*Adlib***
Glucose (mg/dL)	132.8±3.4 ^x^	149.3±3.8 ^y^	135.6±4.1 ^x^
Insulin (ng/mL)	1.08±0.14 ^x^	1.30±0.20 ^y^	1.16±0.15 ^x^, ^y^
HOMA-IR	0.35±0.05 ^x^	0.49±0.08 ^y^	0.40±0.05 ^x^
Total cholesterol (mg/dL)	85.2±4.4 ^x^	99.0±4.9 ^y^	68.9±5.2 ^x^, ^b^
HDL cholesterol (mg/dL)	26.0±1.4 ^x^	32.1±1.6 ^y^	24.1±1.7 ^x^
Triglycerides (mg/dL)	67.5±37.8 ^b^	51.5±44.0 ^b^	54.0±18.0 ^b^

Data are expressed as mean ± SEM except for triglycerides (levels were asymmetric and therefore data was log transformed and expressed as median and interquartile range). ^x,y, a,b^ Values labeled with the same letter are statistically similar and different letters refer to statistical difference by Tukey *post hoc*.

^x,y^ groups comparison

^a,b^ sex comparison (compare tables 2 and 3).

Total cholesterol showed an interaction between group and sex [F (2, 44) = 4.882, p = 0.012], in which males had higher cholesterol levels than females only in the HF_Adlib group (Tukey’s test, p = 0.003). A group effect alone was also observed [F (2, 44) = 6.498, p = 0.003], in which the FR_Adlib group had higher total cholesterol levels than the Adlib_Adlib (Tukey’s test, p = 0.017) and HF_Adlib (Tukey’s test, p = 0.007) groups. There was no sex effect [F (1, 44) = 1.529, p = 0.223].

The analysis of HDL cholesterol showed a group effect [F (2, 44) = 9.071, p = 0.001], in which the FR_Adlib group had increased HDL cholesterol in relation to the Adlib_Adlib (Tukey’s test, p = 0.001) and HF_Adlib (Tukey’s test, p = 0.004) groups. No sex effect [F (1, 44) = 0.038, p = 0.846] or group vs. sex interaction [F (2, 44) = 1.482, p = 0.238] were observed.

A sex effect was observed on TGs [F (1, 44) = 64.678, p<0.0001], in which males had higher TG levels than females in all groups. There was no group effect [F (2, 44) = 0.383, p = 0.684] or group vs. sex interaction [F (2, 44) = 0.731, p = 0.487].

### D2 dopamine receptors in the dorsal striatum

Females in the FR_Adlib group had lower levels of D2 dopamine receptors in the dorsal striatum than those in the Adlib_Adlib group (Student t test, t = 2.716, p = 0.032). No difference was observed between HF_Adlib and Adlib_Adlib (Student t test, t = −2.071, p = 0.068) (Fig. 6).

**Fig 6:** D2 receptor levels in the dorsal striatum of females. Adlib_Adlib vs. FR_Adlib (A) and Adlib_Adlib vs. HF_Adlib (B). Data are expressed as mean ± SEM. Student t test showed a difference between Adlib_Adlib and FR_Adlib (*p = 0.032). OD: optical density.

In males, there were no differences between FR_Adlib (OD: 1.44±0.07) and Adlib_Adlib (OD: 1.52±0.37) (Student t test, t = 0.218, p = 0.835), or between HF_Adlib (OD: 1.33±0.09) and Adlib_Adlib (OD: 1.11±0.19) (Student t test, t = −0.958, p = 0.363).

## Discussion

The main objective of our study was to propose an animal model that would reflect the “similarities in the inequalities” phenomenon previously described in humans, in which extremely unequal social conditions had a similar impact on adult health through different biological mechanisms [19,20]. Health outcomes referred to characteristics that could directly (abdominal fat and metabolic disturbances) or indirectly (behavioral differences) have an impact on adult health and/or survival. We hypothesized that animals subjected to food abundance and scarcity during gestation (corresponding to extremes of inequality) would share similar health behaviors in adulthood (engagement in physical activity). Our hypothesis was confirmed, as the phenomenon was observed in early life (birth weight) and persisted into adult life, when its effects were reflected primarily in behavioral measures (physical activity). In addition, differences in striatal D2 receptor levels between the two extreme groups suggest that behavioral programming occurs via different biological mechanisms and is sex specific, as these differences were observed only in females.

Our model of food restriction during gestation was based on the successful intrauterine growth restriction model described by Desai et al. [26], who have established a rat model of maternal undernutrition that results in intrauterine growth-restricted pups with decreased plasma leptin levels. When provided normal nursing, intrauterine growth-restricted newborns demonstrate significantly increased food intake with rapid catch-up growth, which results in adult metabolic syndrome, including obesity, increased percentage body fat, lipid abnormalities, and insulin resistance [26]. In the current study, we also induced intrauterine growth restriction in pups born to dams that received a high-fat diet. In agreement with studies by Dudley et al. [34] and Howie et al. [35], our results showed that high-fat diet during gestation led to a small but significant reduction in male and female pups’ birth weight. Interestingly, both fetal intervention groups (FR and HF), despite being considered “extremes of inequality” in the current study, induced intrauterine growth restriction in a similar manner. This may be considered the first evidence of the “similarities in the inequalities” phenomenon found in this study. In both conditions, fetuses experience a period of nutrient restriction as a result of alterations in placental delivery [24]. Although a similar result was obtained in pups’ birth weight in our study, it is important to note that the HF group had an increased neonatal mortality rate. One could speculate that such high mortality might be the result of diet change on gestational day 10, although previous studies introducing the high-fat diet before conception have also reported a 50% reduction in pup survival in the HF group [36,37]. According to Shaw et al. [36], the cause of this excess mortality is still unclear.

Regarding pups’ body weight gain and abdominal fat deposition, no significant differences were found between groups. This result contrasts with previous studies reporting increased body weight and abdominal adiposity in animals exposed to intrauterine growth restriction [26,38]. Nevertheless, previous studies of maternal high-fat feeding have provided conflicting results on body weight and abdominal adiposity [39–41], which hinders comparison between studies. This may be explained by the different gestational high-fat protocols applied and/or different post-weaning diets. In the current study, we expected to find the “similarities in the inequalities” phenomenon in these metabolic measures, but this was not confirmed. However, this lack of difference in fat mass between groups should be addressed. Firstly, only abdominal fat from the two major fat depots was weighed, and measurement of body fat content as a whole might have produced different results between groups according to data reported in previous studies [26,38,40]. Secondly, in order support the study hypothesis and main objective, our cohort was young and no “second hit” challenge (e.g. chronic exposure to high-fat diet in adulthood) was applied [42]; these interventions could have increased the odds to elicit differences in fat mass content between groups. Finally, data variation may have prevented us from eventually finding differences that might have been apparent with a larger sample size.

Regarding physical activity, the “similarities in the inequalities” effect could be observed in males from the extreme groups (FR_Adlib and HF_Adlib), which showed significantly less activity than males in the Adlib_Adlib group in some time intervals. These findings reflect the classical developmental origins of health and disease (DOHaD) concept and are in agreement with another study in rodents [42]. These results also provide further evidence to support the view that intrauterine growth restriction establishes a metabolic pattern to save energy (“thrifty phenotype”) [43], a concept that can be expanded to behavioral components (sedentary behavior, increased consumption of palatable foods [44]) or “thrifty behavior” [45]. The “similarities in the inequalities” effect was also observed in females, in which the extreme groups (FR_Adlib and HF_Adlib) were significantly more active than the Adlib_Adlib group in one of the time intervals. It is worth noting that the “similarities in the inequalities” phenomenon in females (increased activity) was the opposite of that in males (decreased activity). While the thrifty phenotype is also described in females in the literature, organs/systems/neural pathways are differentially affected by fetal events in males vs. females, leading to different metabolic disarrangements and behavioral phenotypes. Therefore, although both sexes may be programmed, it is not surprising for us that the effect on physical activity is sexually dimorphic as we demonstrated here.

Interestingly, several studies have proposed that voluntary physical activity in the running wheel is a highly rewarding type of behavior for laboratory rodents [46–52]. Rats demonstrate conditioned place preference to the running wheel associated side [53], and will bar press to have access to the wheels [54–57]. Within this context, alterations in the mesolimbic system could be a possible mechanism to explain the “similarities in the inequalities” effect observed in physical activity. For this purpose, D2 receptors in the dorsal striatum were assessed and showed differences between groups, mostly in females. FR_Adlib had lower D2 receptor levels than Adlib_Adlib, while HF_Adlib did not differ from Adlib_Adlib females. Even though the difference between HF_Adlib and Adlib_Adlib females is not statistically significant, the trend (p = 0.068) is quite interesting, particularly because of the opposite direction of the change in D2 levels when comparing to differences seen between FR_Adlib and Adlib_Adlib females. This suggests that extremely unequal groups (HF_Adlib and FR_Adlib) demonstrate similar behavioral outcomes but by different mechanisms, as discussed below. Further studies exploring this aspect are warranted.

Striatal D2 receptor levels may be important in mediating downstream behavioral responses, including voluntary activity. In the striatum, D2 receptors exert inhibitory control over the firing of medium spiny neurons specifically from the indirect pathway [58]. When there is downregulation of D2 receptors, these neurons are stimulated, impairing motor function and inducing a negative affective state [58]. Surprisingly, in our study, the same group that showed increased levels of spontaneous wheel-running activity also had decreased striatal D2 receptor levels (FR_Adlib females). However, we cannot rule out that D2 receptor downregulation occurs in response to an increased dopaminergic activity in this area in these animals. A recent study has shown that repeated activation of D2 receptors in striatal medium spiny neurons increases the vulnerability to stress-induced depressive-like behavior [59], which may suggest that D2 is more closely related to the emotional motivation for engaging in physical activity than to the motor function itself. Thus, because of decreased D2 receptors, FR_Adlib females would have increased motivation for running in the wheels.

The lack of difference in D2 receptors levels between HF_Adlib and Adlib_Adlib groups confirmed our previous hypothesis, regarding the “similarities in the inequalities” phenomenon that extremely unequal groups, by different mechanisms, would end up with similar behavioral and/or clinical phenotypes. It remains to be defined which mechanism has altered physical activity levels in the HF_Adlib group. This is in agreement with the study by Grissom et al. [60] reporting opposing effects of gestational protein restriction (model of small for gestational age) and gestational high-fat consumption (model of large for gestational age) on the expression of various dopamine-related genes in mesocorticolimbic regions, with substantial similarities in some behavioral outcomes. Likewise, the lack of difference in D2 receptors levels between groups in males suggests that the behavioral sexual dichotomy observed in physical activity in this study has a diverse neural basis. This proposition would be in agreement with a previous study showing dichotomous outcomes between males and females regarding voluntary exercise. In males, voluntary exercise can reduce anxiety-like and depressive-like symptoms, while in females it appears to induce stress [61].

Although no differences were found in body weight and abdominal adiposity in this study, the analysis of biochemical measurements yielded an interesting result. The FR_Adlib group had significantly higher glucose, insulin, insulin resistance (assessed by HOMA-IR) and total cholesterol levels than the Adlib_Adlib group. These findings are consistent with Barker’s hypothesis [62] that people who face adverse intrauterine and/or childhood conditions (such as intrauterine growth restriction) are at increased risk of developing coronary heart disease and diabetes. Other researchers have also confirmed this hypothesis by reporting associations between low birth weight and higher total cholesterol levels in adulthood [63], as well as intrauterine growth restriction and diabetes in men [64,65]. In spite of the fact that our objective was to evaluate “similarities in the inequalities” effects, but our results showed no biochemical differences between HF_Adlib and Adlib_Adlib groups. As discussed above, it is possible that prenatal interventions affect behavioral responses first, and more profound biochemical differences will become apparent only after aging or “second hit” challenges (such as chronic high-fat diet exposure in adulthood).

It is important to point out that there is evidence showing that cross-fostering itself can affect the metabolic phenotype [66]. However, in our study, all experimental groups were subjected to this procedure, and the eventual differences found between groups are, therefore, likely to have resulted from their fetal experience rather than from the cross-fostering procedure.

Our findings showed that the most unequal groups, representing the two extremes of social inequality (maternal undernutrition and overnutrition, respectively, in this study), had the same low birth weight with corresponding behavioral alterations in adult life, similar to what had been previously described in humans [19]. Nevertheless, the “similarities in the inequalities” had an effect mainly on behavioral data, since adult body weight and abdominal adiposity were not affected by this phenomenon. It is possible, as mentioned above, that the animals were too young or that the phenomenon itself is more closely related to behavioral responses. It is important to highlight that it was not the intention of the authors to propose a simplistic animal model for high and low socioeconomic status in humans by manipulating the macronutrient/caloric content of the rat chow per se. We acknowledge the fact that humans have a very complex interaction with their environment and that animal models are not able to fully capture that. For instance, it is known that energy-dense, nutrient-poor foods are preferentially consumed by persons of lower socioeconomic status [67]. However, our model explored the idea of caloric insufficiency versus abundance aiming to represent extreme conditions of a population. Interestingly, we were able to obtain results that resemble the phenomenon previously reported in humans, in which individuals at both ends of the socioeconomic status/birth weight spectrum behaved similarly regarding physical activity [19]. This similar behavior appears to occur through different biological mechanisms considering the differences found in striatal D2 receptor levels between FR_Adlib and Adlib_Adlib, but not between HF_Adlib and Adlib_Adlib groups.

## Supporting Information

S1 Dataset Birth weight dataset. (SAV)

S2 Dataset D2 Western blot FR_Adlib dataset. (SAV)

S3 Dataset D2 Western blot HF_Adlib dataset. (SAV)

S4 Dataset Main dataset (physical activity, metabolism). (SAV)

S5 Dataset Gestational dataset. (SAV)
